The article "MicroRNA-410 Suppresses Migration and Invasion by Targeting MDM2 in Gastric Cancer" was retracted in 2022. Reasons: duplicated images; signs of a paper mill; unreliable results or conclusions.

# MicroRNA-410 Suppresses Migration and Invasion by Targeting MDM2 in Gastric Cancer

**DOI:** 10.1371/journal.pone.0104510

**Published:** 2014-08-19

**Authors:** Jianjun Shen, Weina Niu, Ming Zhou, Hongbo Zhang, Jun Ma, Ling Wang, Hongyan Zhang

**Affiliations:** 1 Department of Radiation Oncology, Anhui Provincial Hospital, Hefei, China; 2 Oncology Department, Anhui Cancer Hospital, Hefei, China; H.Lee Moffitt Cancer Center & Research Institute, United States of America

## Abstract

Gastric cancer is one of the most frequent malignancies in tumors in the East Asian countries. Identifying precise prognostic markers and effective therapeutic targets is important in the treatment of gastric cancer. microRNAs (miRNAs) play important roles in tumorigenesis. However, the mechanisms by which miRNAs regulate gastric cancer metastasis remain poorly understood. In this study, we found that the levels of miR-410 in gastric cancer and cell lines were much lower than that in the normal control, respectively, and the lower level of miR-410 was significantly associated with lymph-node metastasis. Transfection of miR-410 mimics could significantly inhibit the cell proliferation, migration and invasion in the HGC-27 gastric cancer cell lines. In contrast, knockdown of miR-410 had the opposite effect on the cell proliferation, migration and invasion. Moreover, we also found that MDM2 was negatively regulated by miR-410 at the post-transcriptional level, via a specific target site with the 3′UTR by luciferase reporter assay. The expression of MDM2 was inversely correlated with miR-410 expression in gastric cancer tissues, and overexpression of MDM2 in miR-410-transfected gastric cancer cells effectively rescued the inhibition of cell proliferation and invasion caused by miR-410. Thus, our findings suggested that miR-410 acted as a new tumor suppressor by targeting the MDM2 gene and inhibiting gastric cancer cells proliferation, migration and invasion. The findings of this study contributed to the current understanding of these functions of miR-410 in gastric cancer.

## Introduction

Different strategies have been used to treat gastric cancer (GC), which is the fourth most prevalent cancer and the second leading cause of cancer fatalities in the world [1] [2]. Most GC patients is diagnosed at stage III or IV, and the rate of lymph node metastasis is high [3], [4]. Nowadays, patients with the late-stage GC are with an overall 5 year's survival of appoximately 20%[5]. Therefor, it is of great clinical value to further elucidate the molecular mechanisms involved in GC metastasis and to identify novel markers for the diagnosis, prognosis, and the treatment for patients with GC.

microRNAs (miRNAs) are small noncoding RNAs of ∼22 nucleotides in the length that regulate the expression of their target mRNAs through translational repression or mRNA cleavage [6]. They are involved in crucial biological processes, including development and differentiation [7], [8]. The dysregulation of miRNAs is correlated to play an important role in cancer development and progression by regulating the cell proliferation, differentiation, apotosis and carcinogesis [9], [10]. Aberrant expression of miRNAs or mutations of miRNA genes have been well investigated in many types of tumors, including lymphoma, lung, pancreas, leukemia, breast, colon and liver cancers [11]–[15]. However, the roles of miRNAs in GC remain largely unknown.

Previous studies have investigated the role of miR-410 in several cancers. Gattolliat et al [16].demonstrated that the expression of miR-410 was significantly associated with disease free survival of the non-amplified favorable neuroblastoma. Further, Chen at el [17] found that the expression of miR-410 was reduced in human gliomas and forced expression of miR-410 in glioma cells strongly inhibited the cell proliferation, invasion mediated by targeting MET. Moreover, Chien et al [18] found that miR-410 negatively regulated pRb/E2F pathway by directly targeting CDK1 which was an oncogene in breast cancer. However, the role of miR-410 in GC still remains unclear. In this study, we demonstrated that decreased miR-410 expression is a characteristic molecular change in GC and investigated the effect of modulated miR-410 levels on the phenotypes of GC cell lines. We also showed that miR-410 may function as an oncogene by directly targeting MDM2.

## Materials and Methods

### Ethics Statement

All of these patients agreed to participate in the study and gave written informed consent. Both this study and consent were approved by the ethical board of the Anhui Provincial Hospital and complied with the Declaration of Helsinki.

### Human samples

Human GC and their corresponding non-tumorous gastric samples were collected at the time of surgical resection from the Anhui Provincial Hospital from 2008 to 2009. Written informed consent was obtained before collection. One part was fixed with 10% formalin for histopathological diagnosis, and the other was immediately snap-frozen in liquid nitrogen and stored at −196°C in liquid nitrogen until RNA was extracted. Use of human tissues was approved by the Clinical Research Ethics Committee of Anhui Provincial Hospital.

### Cell culture

SGC-7901, HGC-27, MGC-803, MKN-45 and HEK293T cells were purchased from the Shanghai Institute of Biochemistry and Cell Biology at the Chinese Academy of Sciences. Gastric epithelial-1 cell (GES) was obtained from the Shanghai Ruijin Hospital of Shanghai Jiaotong University School of Medicine. The SGC-7901, HGC-27, MGC-803, MKN-45 and GES were maintained in RPMI1640 and HEK293T was maintained in Dulbecco's modified Eagle's medium media. Media was supplemented with 10% foetal bovine serum. The cells were incubated at 37°C in a humidified chamber containing 5% carbon dioxide.

### Plasmids and cell transfection

MiR-410 mimic/inhibitor and the controls were purchased from RiboBio (Guangzhou, China). The HGC-27 cells were seeded in six-well plates at 30% confluence one day prior to transfection. Transfection with miR-410 mimic/inhibitor or the controls was performed using Lipofectamine 2000 reagent (Invitrogen, Carlsbad, CA, USA). Transfection complexes were prepared according to the manufacturer's instructions.

### qRT-PCR

For qRT-PCR assays, total RNA was extracted from cells with TRIzol reagent (Invitrogen, Carlsbad, CA, USA). Reverse transcription was performed with the PrimeScript RT reagent Kit with gDNA eraser (Takara) according to the manufacturer's instructions. The expression of miR-410 was verified by the altered stemloop RT-PCR with specific RT and PCR primers. U6 snRNA was used as an endogenous control. RT reactions were carried out by using RNA fraction with Promega RT Kit following the manufacturer's protocol. The PCR conditions were performed by denaturing the DNA at 94°C for 4 min, followed by 40 cycles of amplification: 94°C for 40 s, 52°C for 40 s, 72°C for 40 s for data collection. Quantitative PCR was performed on an ABI 7500 thermocycler (Applied Biosystems) using SYBR Premix Ex Taq (Perfect Real Time) Kits (TaKaRa, Japan) according to the manufacturer's instructions.

### Cell Proliferation Assay

A total of 10^4^ cells per well were plated in 96-well plates before transfection and cultured for 24 h in normal conditions. They were then transfected with miR-410 mimic or anti-miR-410 inhibitor along with paired negative controls. Cell proliferation was assessed using the Cell Counting Kit 8 (Dojindo, Tokyo, Japan) according to manufacturer's protocol.

### Cell migration and invasion assay

For the migration assays, 5×10^4^ cells were added into the upper chamber of the insert (BD Bioscience, 8-µm pore size). For the invasion assays, 1×10^5^ cells were added into the upper chamber of the insert precoated with Matrigel (BD Bioscience). In both assays, cells were plated in medium without serum, and medium containing 10% FBS in the lower chamber served as chemoattractant. After several hours of incubation, the cells that did not migrate or invade through the pores were carefully wiped out with cotton wool. Then the inserts were stained with 20% methanol and 0.2% crystal violet, imaged, and counted with an IX71 inverted microscope (Olympus).

### Western blot analysis

Proteins were separated on SDS-polyacrylamide gel electrophoresis and transferred to the nitrocellulose membrane (Bio-Rad, Hercules, CA, USA). The membrane was blocked with 5% non-fat milk and incubated with the rabbit anti-MDM2 monoclonal antibody (1∶1000; Cell Signaling Technology, Danvers, MA, USA) and the mouse anti-b-GAPDH monoclonal antibody (1∶10000; Sigma). The proteins were detected with enhanced chemiluminescence reagents (Pierce, Rockford, IL, USA).

### Luciferase reporter assay

HEK293T cells were plated into 96-well plates. After 24-h incubation, a mixture of 100-ng pLUC 3′UTR, 5-pmol negative control, miR-410 mimic was cotransfected with 20 ng.

Renilla into HEK293T cells using Lipofectamine 2000. Forty-eight hours after transfection, firefly and Renilla luciferase activities were measured with the Dual-Luciferase Reporter System (Promega, Madison, WI, USA). The transfection efficiency was normalised by cotransfection with a Renilla reporter vector.

### Statistical analysis

Data were presented as the means ± standard deviation of at the least three experiments. Statistical analysis was performed using SPSS 15.0. A one-way analysis of variance (ANOVA) test and Student's t test were used for statistical analysis. A value of p<0.05 was considered to indicate a statistical analysis.

## Result

### Expression of miR-410 was significantly down-regulated in GC cell and tissue

To assess the role of miR-410 in GC, we evaluated the expression of miR-410 in GC cell line, tissues and their matched normal tissues using quantitative RT-PCR. We found that miR-410 levels were frequently down-regulated in GC cell lines compared with GES. Figure 1B shows that the miR-410 levels were down-regulated in GC tissues compared with those in matched normal tissues. The average expression level in carcinoma tissues (combination) was significantly higher compared with their adjacent non-neoplastic tissues (Figure 1C). We also showed that the expression of miR-410 in the metastases GC tissues was lower than that in non-metastases tissues (Fig. 1D).

**Figure 1:** miR-410 was downregulated in gastric cancer. A. qRT-PCR analysis of miR-410 expression in four cell lines derived from gastric cancer and one nonmalignant gastric cell line (GES). (B) qRT-PCR analysis of miR-410 expression in 60 pairs GC tissues and their corresponding adjacent nontumorous tissues. The expression of miR-410 was normalized to U6 snRNA. (C) Relative miR-410 expression levels in GC tissues and adjacent normal regions; (D) Statistical analysis of the association between miRNA level between pM stage (No metastasis and Metastasis, respectively); *p<0.05, and **p<0.01.

### miR-410 inhibited GC cell proliferation, migration and invasion

The levels of miR-410 were significantly increased in GC cells that were transfected with miR-410 mimics and the miR-410 levels were decreased that were treated with the miR-410 inhibitor (Fig. 2A). Up-regulation of miR-410 inhibited GC cell proliferation; in contrast, knockdown of miR-410 had the opposite effect on the cell proliferation (Fig. 2B). Moreover, the transwell assay and invasion assay showed that the migrated and invasiveness of cells transfected with miR-410 mimics was dramatically decreased compared with the control and untreated cells. We also showed that the migrated and invasiveness of cells transfected with miR-410 inhibitor was dramatically increased compared with the control and untreated cells. (Fig. 2C and D).

**Figure 2:** Overexpression of miR-410 inhibited the cell proliferation, migration, and invasion in gastric cancer cells (A) Expression levels of miR-410 were examined by qRT-PCR after transfection of 20 nmol/L of miR-410 mimics, inhibitors or sramble or no transfection. The expression of miR-410 was normalized to U6 snRNA. (B) The cells treated with miR-410 mimics, inhibitors or sramble or no transfection were measured by CCK8 assay at different time periods. (C) Transwell analysis of HGC-27 cells after treatment with miRNA mimics, inhibitors or scramble or no transfection; the relative ratio of migrated cells per field is shown below. (D) Transwell analysis of HGC-27 cells after treatment with miRNA mimics, inhibitors or scramble or no transfection; the relative ratio of invasive cells per field is shown below, *p<0.05, ** p<0.01, and ***p<0.001.

### miR-410 directly targeted MDM2 in GC

As predicted by PicTar, there was complementarity between has-miR-410 and MDM2 3′-UTR (Fig. 3A). To demonstrate that miR-410 directly regulates MDM2, we employed a dual-luciferase reporter system. We found that co-expression of miR-410 significantly suppressed the firely luciferase reporter activity of the wild-type MDM2 3′UTR but not the mutant 3′UTR (Fig. 3B). Overexpression of miR-410 reduced the expression of MDM2 mRNA and protein (Fig. 3C and D).

**Figure 3:** miR-410 targets at MDM2 in GC cells. (A) The sequences of miR-410 binding sites within the human MDM2 3′UTRs and schematic reporter constructs, in this panel, c-MDM2-WT represent the reporter constructs containing the entire 3′UTR sequences of MDM2. C-MDM2-MUT represent the reporter constructs containing mutated nucleotides. (B) The analysis of the relative luciferase activities of MDM2-WT, MDM2-MUT in 293T cells. The error bars are derived from triplicate expriments. (C) qRT-PCR analysis of MDM2 mRNA expression in HGC-27 cells after treatment with miRNA mimics or scramble or no transfection. The expression of MDM2 was normalized to GAPDH. (D) Western blot analysis of MDM2 expression in HGC-27 cells transfected with miR-410 mimics or scramble or no transfection. GAPDH was also detected as a loading control.

### Overexpression of MDM2 inpaired miR-410-induced inhibition of invasion in GC cells

We performed rescue experiments by transfection of 3′UTR-negative MDM2 together with miR-410. As expected, transfection with the pcDNA3.1-MDM2 alleviated the reduction of MDM2 resulted from miR-410 mimic treatment (Fig. 4A). In agreement with the expression of target proteins, transfection with the pcDNA3.1-MDM2 mitigated the inhibition of cell amplification (Fig. 4B) and the increase of invasive cells (Fig. 4C) resulted from miR-410 mimic treatment.

**Figure 4:** Overexpression of MDM2 impaired miR-410-induced inhibition of proliferation and invasion in GC cells (A) Western blot analysis of MDM2 in HGC-27 cells co-transfected with either miR-410 mimic or scramble and 2.0 µg pCDNA-MDM2 or pCDNA empty vector. (B) Cell growth curves in HGC-27 cells transfected with different combinations. (D) Transwell analysis of HGC-27 cells treated with different combinations. The relative ratio of invasive cells per field is shown right. *p<0.05, ** p<0.01, ***p<0.001.

### MDM2 was inversely expressed with miR-410 in GC

To further elucidate the relationship between miR-410 and MDM2 expression in primary samples, we firstly detected MDM2 in GC cell lines. As shown in Fig. 5A and 5B, the mRNA and protein expression of MDM2 was much higer in the 4 GC cell lines than that in the GES. We also found that the expression of MDM2 in GC tissues was significant higher than in the corresponding adjacent normal tissues (Fig. 5C). The scatter plot and the Pearson correlation analysis further showed that miR-410 expression was negatively correlated with the target protein levels in the GC samples (Fig. 5D). These data suggested that the decreased miR-410 expression was related to the increased MDM2 levels in the most of the GC patients.

**Figure 5:** miR-410 negatively regulated MDM2 gene expression. (A) The relative MDM2 mRNA expression levels were determined by qRT-PCR in four cell lines derived from gastric cancer and one nonmalignant gastric cell line (GES). The expression of MDM2 was normalized to GAPDH. (B) Western blot analysis of MDM2 expression in four cell lines derived from gastric cancer and one nonmalignant gastric cell line (GES). GAPDH was also detected as a loading control. (C) qRT-PCR analysis of MDM2 expression in 40 pairs gastric cancer tissues and their corresponding adjacent normal tissues. The expression of MDM2 was normalized to GAPDH. The expression of MDM2 in gastric cancer tissues was significant higher than in the corresponding adjacent normal tissues. (D) Analysis of correlation of miR-410 and MDM2 expression in gastric cancer tissues. *p<0.05, ** p<0.01, ***p<0.001.

## Discussion

miRNAs have acted as important regulators of gene expression at the post-transcriptional level and regulate a wide range of physiological and developmental processes [6], [19], [20]. Mounting evidences suggest that alterations in the expression of miRNAs contribute to the pathogenesis of the most human cancers, which they can act as either oncogenes or tumor suppressors [21], [22]. Recently, accumulating data indicate that miRNAs are involved in several important biological events such as tumorigenesis and cancer metastasis [23], [24]. In the present study, we investigated the biological role of miR-410 in human GC tumorigenesis. Our results demonstrated that miR-410 was frequently down-regulated in human GC and that its down-regulation was significantly associated with clinical stage and lymph node metastasis. Enforced expression of miR-410 could increase the proliferation, migration and invasion of the GC cells line in vitro. We further identified MDM2, a putative tumor suppressor gene, as a direct functional target of miR-410. To our knowledge, this is the first study to explore the role of miR-410 in GC, and our results indicated that miR-410 acted as a new oncogene in GC.

Deregulation of miR-410 is a frequent event in various cancers, suggesting that miR-410 may play an important role in tumorigenesis and tumor progression. Gattolliat and colleagues show that miR-410 expression was significantly associated with disease free survival of the non-amplified favorable neuroblastoma [16]. Further, Chen [17] found that miR-410 expression was reduced in human gliomas and forced miR-410 expression in glioma cells strongly inhibited the cell proliferation, invasion mediated by targeting MET. However, the expression and function of miR-410 in GC development has not been reported. In this study, we identified the expression of miR-410 in several GC cell lines and the GES using qRT–PCR. The expression of miR-410 was significantly increased in all four GC cell lines compared with in the GES. Furthermore, the results obtained from clinical GC tissue also confirmed that miR-410 was down-regulated in the GC tissues compared to the paired non-cancerous adjacent tissues, indicating its possible involvement in both oncogenic transformation and tumor metastasis. We subsequently confirmed that inhibition of miR-410 significantly promoted GC cell proliferation, migration and invasion in vitro.

We further explored the molecular mechanism underlying the role of miR-410 and identified MDM2 as a direct functional downstream target of miR-410 in the GC cells. Bioinformatics approaches, which were used to predict targets of miRNAs, highlighted a high free-energy seed match at the well-conserved miRNA-binding site and its target mRNAs, but specificity remained a problem in defining targets of many miRNAs. Thus, over-expression of a miRNA could down-regulate the expression of the target protein. Complementary sequence of miR-410 is identified in the 3′UTR of MDM2 mRNA. Further, we demonstrated that miR-410 directly targets the 3′UTR of MDM2, as its overexpression was associated with suppression of luciferase activity. In addition, a significant down-regulation in the level of MDM2 protein was observed after miR-410 overexpression, indicating posttranscriptional regulation of MDM2 via targeting its 3′UTR. These results indicated that miR-410 may function as a tumor suppressor partly mediated by repressing miR-410 expression in GC development.

MDM2 is an oncogene that was firstly discovered in a locus amplified on double minute chromosomes in a tumorigenic mouse cell line (3T3-DM) [25]. The main function of MDM2 is to inhibit p53 bioactivity by blocking the transcriptional activity of p53 and promoting p53 protein degradation [26]–[28]. High MDM2 levels decreased p53 protein levels and can attenuate p53 function, which increased cancer risk and/or accelerated tumor formation and progression [29]. The MDM2 oncogene played an important role in cancer progression [30]. Overexpression of MDM2 in tumor cells induced cell proliferation, inhibits cell apoptosis [31]. Several studies have showed that MDM2 overexpression was associated with poor survival and was a useful predictive factor for poor prognosis in humans with hepatocellular carcinoma and breast carcinomas [32], [33]. Moreover, the recent study have found that MDM2 was expressed at higher levels in GC tissues than in non-cancerous gastric mucosa, and MDM2 expression was associated with clinicopathologic features in patients treated only with surgery [34], [35]. Moreover, knockdown of MDM2 or overexpression of JWA has the synergistic effect on suppression of gastric cancer cell proliferation and migration [35]. However, the mechanism how MDM2 was overexpression is still unknown. These results indicated that the ability of miR-410 to target MDM2 may provide one such mechanism of post-transcriptional control of MDM2.

In summary, our results have showed that miR-410 was significantly down-regulated in GC cells and tissues. Enforced expression of miR-410 increased GC cell proliferation, migration and invasion through directly targeting MDM2. These findings suggest that this novel miR-410/MDM2 axis provides new insight into the mechanisms underlying tumor metastasis, and repression of miR-410 expression may be a potential therapeutic strategy for the treatment of GC in the future.

## Supporting Information

Table S1 **Clinicopathologic charateristics of patients with GC.**
(DOCX)

Table S2 **Primer sequence.**
(DOCX)
